The article "Artificial Intelligence-Based Data-Driven Strategy to Accelerate Research, Development, and Clinical Trials of COVID Vaccine" was published in 2022. Journal: Biomed Res Int.

# Artificial Intelligence-Based Data-Driven Strategy to Accelerate Research, Development, and Clinical Trials of COVID Vaccine

**DOI:** 10.1155/2022/7205241

**Published:** 2022-07-06

**Authors:** Ashwani Sharma, Tarun Virmani, Vipluv Pathak, Anjali Sharma, Kamla Pathak, Girish Kumar, Devender Pathak

**Affiliations:** ^1^School of Pharmaceutical Sciences, MVN University, Haryana 121102, India; ^2^GL Bajaj Institute of Technology and Management, Greater Noida, Uttar Pradesh, India; ^3^Freelancer, Pharmacovigilance Expert, India; ^4^Uttar Pradesh University of Medical Sciences, Etawah, Uttar Pradesh 206001, India; ^5^Rajiv Academy for Pharmacy, NH. #2, Mathura Delhi Road P.O, Chhatikara, Mathura, Uttar Pradesh 281001, India

## Abstract

The global COVID-19 (coronavirus disease 2019) pandemic, which was caused by the severe acute respiratory syndrome coronavirus 2 (SARS-CoV-2), has resulted in a significant loss of human life around the world. The SARS-CoV-2 has caused significant problems to medical systems and healthcare facilities due to its unexpected global expansion. Despite all of the efforts, developing effective treatments, diagnostic techniques, and vaccinations for this unique virus is a top priority and takes a long time. However, the foremost step in vaccine development is to identify possible antigens for a vaccine. The traditional method was time taking, but after the breakthrough technology of reverse vaccinology (RV) was introduced in 2000, it drastically lowers the time needed to detect antigens ranging from 5–15 years to 1–2 years. The different RV tools work based on machine learning (ML) and artificial intelligence (AI). Models based on AI and ML have shown promising solutions in accelerating the discovery and optimization of new antivirals or effective vaccine candidates. In the present scenario, AI has been extensively used for drug and vaccine research against SARS-COV-2 therapy discovery. This is more useful for the identification of potential existing drugs with inhibitory human coronavirus by using different datasets. The AI tools and computational approaches have led to speedy research and the development of a vaccine to fight against the coronavirus. Therefore, this paper suggests the role of artificial intelligence in the field of clinical trials of vaccines and clinical practices using different tools.

## 1. Introduction

Virus-caused infectious diseases have long been the most difficult challenge in human health. High-infectivity and high-mortality diseases are particularly feared, and in the past, people viewed them as a tragedy or disasters (Hilleman et al., [1]). Humankind has been able to overcome the irrational dread of death because of advances in recognizing the etiology of viral diseases and knowledge of microbiology, which were followed by the creation of numerous vaccines. Vaccination is often regarded as one of the greatest achievements in medical history. Immunization has saved a lot of lives, and its significance continues to expand. Despite countless efforts to develop qualified and efficient vaccinations, there are inadequate barriers in place to protect populations from diseases that could produce epidemics or pandemics (for example, the Ebola virus epidemic) (Kilbourne, [2]; Gostin et al., [3]). As a result, scientists are working to expand the viral infection that may be prevented by vaccinations, as well as the population groups that will benefit from vaccination in the long term. As of now, Coronaviruses (CoVs) are responsible for the causes of serious illnesses in humans and a variety of animal hosts, including respiratory, gastrointestinal, and systemic diseases. Infections with the CoVs have been found in cattle, swine, rats, cats, mink, dogs, bats, palm civets, horses, camels, ferrets, rabbits, snakes, and a variety of other wild mammals and bird species (Fehr and Perlman [4], Kahn and McIntosh, [5]). Since the very first outbreak in 2002, the Coronaviridae virus family, which causes pneumonia-like symptoms, has been a global danger (Khan et al., [6]). The infections including severe acute respiratory syndrome (SARS) and middle eastern respiratory syndrome (MERS), which first occurred in 2002 and 2013, respectively, caused respiratory and gastrointestinal problems (Hilgenfeld and Peiris, [7]). SARS-COV-2, which has been identified as the virus that causes COVID-19, having symptoms ranging from a common cold to serious respiratory failure, was the source of a third coronavirus episode in 2019 (Kong et al., [8]). Compared to the World Health Organization's (WHO) declaration of a pandemic, COVID-19 has started spreading and has affected at least 20 million people, with a mortality toll of around 5 lakh at the time of such an assessment (Worldometer, [9]). Due to the inadequacy of lab-based high throughput screening (HTS), virtual screening (VS) has emerged as a preferred tool for discovering effective molecules while hospitals continue to trial and error strategies for COVID-19 drug discovery (Jin et al., [10]; Kandeel and Al-Nazawi, [11]). The strategy of specifically targeting biomolecule (e.g., DNA, protein, RNA, and lipid) by using a computer program, of a cell to suppress its growth and/or activity is known as rational drug discovery which can be recognized by VS (Shoichet, [12]; Lionta et al., [13]). Two significant subgroups of this form of screening are ligand-based and structure-based drug design and discovery (Lionta et al., [13]; Yu and Mackerell, [14]; KeshavarziArshadi et al., [15]). Computationally and experiment-based access can determine the viral protein structures and antiviral candidates can be identified quickly and at a low cost using VS (Senior et al., [16]; Zhang et al., [17]). Furthermore, traditional vaccine development approaches are expensive, and developing an effective vaccine against a specific virus might take many years. COVID-19 vaccines have been developed and manufactured with much effort, and the efforts to advance vaccine clinical trials have been tremendous. Coronaviruses are positively stranded RNA viruses that have their genome packaged into the nucleocapsid (N) protein and are surrounded by the membrane (M), envelope (E), and spike (S) proteins (Li, [18]). While many coronavirus vaccine experiments targeting various structural proteins were done, most of these efforts came to an end soon after the SARS and MERS outbreaks. The first human trial of the mRNA-based vaccination targeting the SARS-CoV-2's S protein began on March 16, 2020, as an expedient response to the COVID-19 pandemic. S protein is the coronavirus's most superficial and protrusive protein, and it plays a critical function in the entry of the virus. Because of their capacity to induce neutralizing antibodies that block host cell entry and infection, the full-length S protein and its subunit S1 (which contains the receptor-binding domain) have frequently been employed as vaccine antigens in the development of SARS and MERS vaccines. Current coronavirus vaccines, particularly S protein-based vaccines, may, however, have challenges with producing complete protection and potential safety concerns (Roper and Rehm, [19]; De Wit et al., [20]).

Nonetheless, sterile immunity and full protection are desired outcomes of a COVID-19 vaccine. Furthermore, it is becoming increasingly obvious that diverse immune responses, such as those elicited by cell-mediated or humoral immunity, are more important predictors of protection than antibody titers alone (Ong et al., [21]). One of the technology reverse vaccinology (RV), which is aimed at uncovering viable vaccine candidates through bioinformatics analysis of the pathogen genome, has transformed vaccine research in recent years.

## 2. Reverse Vaccinology

Reverse vaccinology (RV) was introduced in the early 1990s as a genome-based vaccine design approach (Rappuoli, [22]; Bullock et al., [23]) and attributed to the reason that bacterial culturing was no longer needed for selecting vaccine targets; the field was transformed to a more efficient status (Soria-Guerra et al., [24]; Heinson et al., [25]; Bruno et al., [26]). Its goal is to use bioinformatics to analyze the pathogen genome to find a good vaccination candidate. RV has been used to develop vaccines against infections like Group B meningococcus, which resulted in the approval of the Bexsero vaccine (Folaranmi et al., [27]). The research and application of vaccine-like compounds to humans date back to prehistoric times. Hilleman et al. drew a simple diagram to show this history (Figure 1). We are living in the present era of vaccine development, which is more effective and productive than any previous period in history, according to this diagrammatic overview. This advancement has been achieved due to generous financial support as shown in Figure 1 (Hilleman et al., [1]).

In recent decades and for future perception, AI is the most emerging and demanding scientifically engineered technique. Through this, the computational understanding of machines can be obtained by incorporating intelligent behavior to innovate intelligent and smart machines. AI consists of various pieces of techniques, tools, and algorithms such as neural networks, symbolic AI, deep learning, machine learning, and genetic algorithms. These tools are growing and showing impact in different fields like military, space, robotics, and health. AI term was given by John McCarthy while he was at a conference on this subject in 1956 (McCarthy, [28]; Turing, [29]; Russell et al., [30]). In recent years, the advanced featuring tool of AI is machine learning (ML) reorganized in different fields of engineering and science. Nowadays, it is largely adopted in our daily lives, but the ability to find out the conceptual abstract from the large volume of data and feature learning is the most powerful contribution of ML as a tool of AI (Lecun et al., [31]; Grover and Toghi, [32]; Sun et al., [33]). The subbranches of AI are depicted in Figure 2.

AI is applied to medicine and has two main divisions, which are virtual and physical; the virtual part is acted by ML (also called deep learning), and its representation is achieved by mathematical algorithms, as a count of its experience; it improves learning. Based on ML algorithms, there are three divisions:

1. Supervised (prediction and classification algorithms based on former examples)
2. Unsupervised (patterns finding ability)
3. Reinforcement learning (rewards sequences and punishments are used to build a scheme for operation in a particular problem)

Earlier, AI has raised and is still raising the impact of its techniques in genetics and molecular medicine discoveries due to algorithms of machine learning and management of knowledge. A great example of success in the development of medicine and vaccine is determined by unsupervised protein-protein interaction algorithms, which can lead to remedial target discoveries (Theofilatos et al., [34]). Adaptive evolutionary algorithms and state-of-the-art clustering are the two methods used in the combination and that novel methodology is named “evolutionary enhanced Markov clustering.” More than 5000 protein complexes are under this permitted prediction from which at least one gene ontology function phrase reinforced over 70% of the results. The development of a novel computational methodology is permitted to identify single-nucleotide polymorphisms (SNPs) of DNA variants to predict the traits or diseases by employing revolutionary evolutionary. This works by embedding algorithms that are more robust and less prone to over-fitting problems that occur when a model has too many parameters with the number of observations (Rapakouliaet al., [35]; Theofilatos et al., [34]). According to the predictions, the most effective method for drug development is the Graph Convolution Neural Network (GCNN) (Duvenaud et al., [36]; Kearnes et al., [37]). These networks can retain graphs and extract properties from the information encoded within the compound characteristics. AI contributes to learning which can be successfully done by GCNN for a molecule and compound's prediction such as property and protein interface estimation (Fout et al., [38]; Liu et al., [39]). Some models are sequence-based like proteomics, transcriptomics, and genomics. They have shown an impact in recent years because of natural language processing (NLP) domain advancement, but more advanced generation models are context-based models which gain the attention from sequence-based models (Devlin et al., [40]).

Furthermore, vaccine development techniques are being adapted to certain countries' economic and health needs. This tendency has a direct impact on the goods in development as well as the quantity and types of clinical studies conducted. This chapter briefly summarizes the role of AI-based models in COVID-19 drug discovery or research and vaccine development (clinical trials). It is to be proposed that a concentrated effort be made to use AI methodologies to utilize information from preexisting data.

### 2.1. Coronavirus Structure

Coronavirus's basic structure is made up of five proteins, which are named as follows: spike proteins (S), Membrane proteins (M), envelope glycoproteins (E), nucleocapsid proteins (N), and hemagglutinin esterase (HE). Spikes are thought to have three heads (S1) and a trimeric stalk, according to several studies (S2). S1 connects to a host cell's particular surface receptors for viral attachment, whereas S2 binds to the viral and host membranes at the time of virus penetration. This makes it possible for the virus to infect the cells of the host (Li, [18]). The structural proteins are M proteins that aid in the determination of a virus's shape (Neuman et al., [41]). These are the most common proteins in CoVs. These proteins are primarily responsible for RNA packing (Tang et al., [42]). The protein E is extensively produced inside the infected cell during the replication cycle (Venkatagopalan et al., [43]). Furthermore, E protein is involved in viral budding, assembly, and morphogenesis (Nieto-Torres et al., [44]). Phosphoproteins with the ability to attach to the RNA genome are known as N proteins (de Haan and Rottier, [45]). The N protein is required for virion assembly, replication, and CoVs transcription. It aids in the budding and assembly of viruses (Tooze et al., [46]). Certain enveloped viruses have a glycoprotein called HE. The host cell surface receptor is a sialic acid derivative, and HE aids in its adhesion or recognition. It is the one who is responsible for the receptor's demise (de Groot, [47]; Zeng et al., [48]).

### 2.2. COVID-19: Molecular Mechanisms and Target Selection

The spikes on the coronavirus bind to a receptor present on the surface of a cell. After fusing with the cell membrane, the virus releases its RNA genome into the cell. The cell then produces copies of RNA as well as structural proteins required for the assembly of new virus particles, which are then discharged into the body. The role of the immune system is to destroy pathogens such as bacteria and viruses that are causing disease. Its first step is an innate immune response that is to send a variety of weapons to fight infection. But if the pathogens are new to the body and this response does not work to fight infection then, an adaptive immune response comes into action. During the adaptive immune response, specialized cells envelop the virus and deliver antigens, which activate immune cells. The two types of white blood cells are B cells and T cells which play a role in adaptive immunity. Antibodies are specialized proteins that are produced by B cells that bind to pathogens and prevent them from infecting healthy cells. T cells can destroy virus-infected cells that prevent them from replicating the virus. Meanwhile, memory B and T cells record the antigens, ensuring that the body responds rapidly if the coronavirus encounters again (Waltz, [49]). B cells are important in humoral immunity because they can secrete antibodies that neutralize the antigen. The ElliPro web tool (http://tools.iedb.org/ellipro/) was used to forecast both discontinuous and linear B cell epitopes. B cell epitopes assist in the detection of viral infections in the immune system. At the 0.51 threshold, ABCpred (http://crdd.osdd.net/raghava/abcpred/) was utilized to forecast 14-mer B cell epitopes for target proteins (Saha and Raghava, [50]; Ponomarenko et al., [51]; Rafi et al., [52]). T cell epitopes are important in the development of vaccines. It saves money and time as compared to laboratory experiments. 8–11 mer MHC class-I and 11–14 mer MHC class-II epitopes were predicted using the IEDB consensus technique (http://tools.iedb.org/mhcii/) (Zhang et al., [53]; Tahir ulQamar et al., [54]).  Figure 3(a) shows a schematic representation of adaptive immunity targeting pathogens for killing.

### 2.3. COVID-19: Vaccines

A vaccine usually contains an agent that looks like a disease-causing germ (microorganism) and is manufactured from weakened or destroyed microbes, one of their surface proteins, or their toxins. The agent induces the body's immune system to detect the agent as a threat as well as any microbes connected with it (Melief et al., [55]; Bol et al., [56]). Vaccines can be used as preventive or therapeutic measures (Brotherton, [57]; Frazer, [58]). Vaccines are the most significant public health measure against COVID-19 around the world as SARS-CoV-2 is a highly contagious virus infecting people all over the globe (Amanat and Krammer, [59]).  Figure 3(b) shows the role of the vaccine in preventing the spread of a virus. COVID-19's spread shows no signs of halting, and its fatality rate is relatively high when compared to other viral-based infections; the development of vaccines and antiviral treatments against SARS-CoV-2 is very critical and essential. Most vaccines take years to develop ranging from 5 years for Ebola and 40 years for polio. On average, vaccines took 15 years. The vaccine trial process consists of various steps that must be followed quantitatively and systematically. The length of this process is proportional to the vaccine's purpose and nature, which is to protect healthy people from pathogen infection (Deb et al., [60]; Thanh Le et al., [61]). As this virus is fatal, our societies and economies are unlikely to return to normal until a highly effective vaccination has been given to a large section of the world's population.

The hunt for a safe and effective vaccine was grown to be a massive project involving thousands of researchers working in laboratories pursuing different platforms for COVID-19 vaccine all over the globe. COVID-19 vaccine development platforms include several novel technologies. Vaccines work by presenting antigens that cause the immune system to respond without getting the individual sick. Vaccines come in a variety of forms, including weakened versions of the complete virus, DNA or RNA, and specific virus fragments that drive a cell to produce a specific virus fragment. The costly and long process of vaccine development can be accelerated using computational methods. However, because of the urgent necessity and deteriorating situation worldwide, some scientists (Pfizer) raced to develop COVID-19 vaccines. The pharmaceutical industry incorporated artificial intelligence in several areas of the development of vaccines and trials during the process. The scientists need to go through each data set for checking errors and other irregularities that occur naturally while collecting millions of data points. Advantageously, technology helped to reduce the effort smoothly. As reported by Cohen in Science magazine [62], the American company Moderna has reduced the time it takes to develop a human-testable vaccine prototype by utilizing bioinformatics technologies in which AI looks to play a crucial role. Moderna was one of the first to introduce a COVID-19 vaccination that was effective. Moderna is also utilizing artificial intelligence to aid in the development of mRNA sequences. Dave Johnson, an AI Officer, and Moderna's Chief Data show how robotic automation and AI algorithms allowed them to go from manually creating roughly 30 mRNAs per month to being able to manufacture over 1,000 per month. Its use of AI to speed up development was one of the reasons it was able to achieve this breakthrough so swiftly (Gast, [63]). AstraZeneca, a major contributor to the COVID-19 vaccine, is employing artificial intelligence not only in the development of the Covishield vaccine but also in drug discovery. AstraZeneca was one of the first companies to use artificial intelligence in the healthcare sector. To make the drug-making method less expensive, safer, and faster, the company has introduced AI into each step of the research and development process. AstraZeneca has combined knowledge graph and image analysis to get new insights into diseases and detect biomarkers 30% faster than human pathologists (Beatrice, [64]). Thermoregulated storage is required for the entirety of COVID-19 vaccinations. Covishield from Oxford-AstraZeneca and Covaxin from Bharat Biotech, for example, demand a storage temperature of 2–8°C. IoT based on sensor technology, which allows for continuous real-time data monitoring, can help to ensure a reliable storage system. If the temperature changes, the sensors will detect it and issue a device alert for the next vaccination shipment (Kumar and Veer, [65]). AI was successfully employed by Pfizer to run vaccine trials and expedite distribution. Pfizer, on the other hand, used AI throughout the vaccine development process to ensure that the COVID-19 vaccine met the needs of individuals. Pfizer began automating its research and development activities and incorporating artificial intelligence into its working system even before the epidemic. The company employed artificial intelligence algorithms to help identify signals amid millions of data points in its 44,000-person research during the vaccine trials. AI was applied in several aspects of vaccine development and trial during the vaccine development process by the pharmaceutical industry. After satisfying the key efficacy case counts, the data were analyzed and made available in approximately 22 hours with the help of an ML tool, i.e., Smart Data Query (SDQ). Throughout the study, the ML technique assured data quality, requiring very little human interaction (Beatrice, [66]).  Table 1 shows the implications of AI/ML in some of the vaccines for SARS-COV-2. Live attenuated, inactivated, and inactivated with adjuvant vaccines are still being developed using the traditional process. Recombinant subunit vaccines as well as more advanced approaches along with DNA and RNA-based vaccines are also being used (Thanh Le et al., [61]; Zhang et al., [17]; Lurie et al., [67]).

## 3. AI in Vaccine Research

Studying the proteins that make up the virus, such as the spike protein (S), is one of the roles and functions of AI in vaccine development. An AI system can sort through thousands of components in a complicated structure to find the ones most likely to elicit a strong immunological response. To ensure that a vaccine remains effective over time, AI systems must identify components that are unlikely to change or mutate. In the search for a vaccine, a crucial role has been seen for computational analyses and machine learning algorithms. These technologies are helping in assisting researchers in better understanding the virus with its structure and predicting which of its components will elicit an immune response, which is an important and main stage in vaccine development. These techniques can assist researchers in selecting the components for possibly potential vaccines and making sense of experimental data. By merging data from numerous experimental and real-world sources, AI allows scientists to derive insights. They also help in tracking the virus's genetic alteration (mutation) over time, which will determine the value of any vaccine in the future time (Waltz, [49]).

## 4. Different AI Tools

It has been documented that the National Institute of Allergy and Infectious Diseases funded the first clinical trial of an AI-based flu vaccine in 2019 in the United States (Ahuja et al., [71]). Flinders University scientists created the vaccine with the use of an AI tool called synthetic chemist, which generated trillions of synthetic chemical compounds. The researchers next used the Search Algorithm for Ligands (SAM), an AI program that sifts through trillions of molecules to determine which one might be a good vaccine adjuvant candidate (Park, [71]). This method can lessen the time it takes to develop a vaccine by several years. Screening compounds as potential adjuvants for the SARS-CoV-2 vaccine as well as a screening of new compounds based on modeling of probable changes or mutations to the novel coronavirus is easier with an AI-based approach. As the virus is having the potential to mutate, this will aid in the development of vaccines (Ahuja et al., [71]). It has never before been seen in human history for such a race to develop a vaccine against a virus. But by utilizing the power of AI, the velocity of discovery can be greatly enhanced.  Figure 4 shows the process of discovering vaccine candidates via the AI/ML method.

Over the last two decades, machine learning has also aided vaccine development. Machine learning-provided ligand-protein interaction, reaction prediction (Fooshee et al., [72]), activity prediction (Zhavoronkov et al., [73]), and compound property prediction (Ma et al., [74]) are the most affected domains of vaccine and drug discovery (Chen et al., [75]). RV is a technique for developing novel vaccines that begin with pathogen genome sequencing. Through bioinformatics analysis of the pathogen genome, RV tries to identify potential vaccine candidates. By selecting epitopes and screening vaccine candidates in silico, RV can be used to choose an antigen for a novel vaccine that can elicit an immunological response and also speed up and lower the cost of the process of vaccine development (Rappuoli et al., [22]; Mora et al., [76]; Hwang et al., [77]).

VaxiJen was the first application of machine learning in RV methods, and it has shown encouraging antigen prediction outcomes (Doytchinova and Flower, [78]; Heinson et al., [79]). Vaxign, the first web-based RV program (He et al., [80]), has been used to predict vaccine candidates against a variety of viral and bacterial infections (Xiang and He, [81]). Vaxign's first generation uses a filtering-based strategy to choose vaccine antigen candidates based on the user's past knowledge of the pathophysiology of the target pathogen (Ong et al., [21]). Recently, Vaxign-ML, a machine learning approach, has been developed to enhance prediction accuracy (Ong et al., [82]).Vaxign-ML used the biological and physicochemical properties of protein sequences as input variables to train five different machine learning models. The input protein sequences were taken from the Protegen database, which has been collecting and annotating experimentally confirmed protective antigens for the past ten years (Yang et al., [83]; Ong et al., [21]). In a study, data was gathered from the Immune Epitope Database (IEDB), the Virus Pathogen Resource, and the National Center for Biotechnical Information by a team from the University of Southern California. Over 600,000 epitomes from 3,600 distinct species are stored in the IEDB. When applied to SARS-CoV-2, the AI model immediately ruled out 95% of the elements that could be COVID therapies, highlighting the best alternatives. This AI tool predicted a total of 26 possible potential vaccines to combat the deadly infections. The researchers chose 11 of the 26 to use in the development of a multiepitope vaccine that targets the viral spike proteins that are important for replication. The suggested vaccine design framework can address the three most commonly observed mutations and may be expanded to include other potentially unknown mutations. Several vaccines have been in use now, but in case the mutation occurs and possibly reduces the effectiveness of vaccines in use, the AI-assisted method will be able to provide quick results to design other preventive mechanisms. Currently, AI technology only employs B cell and T cell epitopes to generate findings. IgPred is a tool that predicts when immunoglobulin subclass a B cell epitope is capable of. The tool was trained using the support vector machines (SVM) method on over 14,000 epitopes and can be used to detect epitopes that induce IgG and IgA antibodies (Gupta et al., [84]; Khairkhah et al., [85]). NetCTLpan has been used in multiple SARS-CoV-2 vaccine development studies, and it provides end-to-end cytotoxic T cell epitope predictions (Mishra, [86]; Ayyagari et al., [87]). AI technology can create a stronger and faster vaccine if given more datasets and viable combinations. This approach is thought to be capable of accurately predicting over 700,000 distinct proteins (Komarraju, [88]). It is critical to forecast the peptides that bind multiple human leukocyte antigen (HLA) molecules to build and develop an effective vaccine for a large population (Brusic et al., [89]). MHC-I and MHC-II proteins encoded by the HLA gene present epitopes as antigenic determinants. Recursive feature elimination (RFE), SVM, and random forest (RF) are examples of machine learning algorithms that have been used to identify antigens from protein sequences (Bowick et al., [90]; Rahman et al., [91]). Detecting the presence of antigenic peptides presented by MHC-II is one of the most straightforward applications of ML and other AI-based technologies in vaccine development. The examples which can predict antigen presentation are MoDec and MARIA (major histocompatibility complex analysis with recurrent integrated architecture). To better understand natural immunity, various AI-related technologies have been employed to examine SARS-CoV-2 viral peptide presentation on MHC molecules from patients. Thus, it could aid either directly or indirectly in the discovery of COVID-19's unique immune response and the development of a successful vaccine. MARIA improves HLA-II prediction by integrating better training data with a novel supervised machine learning model that uses a multimodal recurrent neural network. (RNN). A similar technique to the convolutional neural network (CNN) is a motif deconvolution technique known as MoDec. It has been used to find out peptide cleavage and MHC-II binding motifs from MS-based peptidome datasets that compromises HLA-DP, HLA-DQ, and HLA-DR alleles. To detect B cell and T cell epitopes of SARS-CoV-2, Fast et al. [92] used two artificial neural network techniques known as MARIA and NetMHCPan4. The technique discovered 405 T cell epitopes with high MHC-I and MHC-II presentation scores, as well as two putative neutralizing B cell epitopes on the S protein. This discovery will aid in the development of effective COVID-19 vaccines and neutralizing antibodies (Racle et al., [93]; Chen et al., [94]; Moore et al., [95]; Arora et al., [96]). A recent study has used a combination of computational techniques and immunoinformatics, thus identifying antigenic epitopes in the structural proteins of SARS-CoV-2 (S, E, M) and suggested a plausible multiepitope-based subunit vaccine (MESV). MESV has sufficient structural and physicochemical characteristics to activate all components of the host immune system. It also seems to have a very stable interaction with the innate immune receptor toll-like receptor-3, making it more likely to enter the host immune system. By the use of computational tools, this study could help researchers save time and money when studying experimental epitope targets (Tahir ulQamar et al., [54]). The development of AI algorithms for determining whether a peptide binds numerous HLA molecules is extremely important in making the design of vaccines more time-efficient. The proposed systems include systems based on hidden Markov models (HMMs), artificial neural networks (ANNs) (Brusic et al., [97]), and SVMs (Bozic et al., [98]). SVM has been used to predict antigens in an RV problem (Heinson et al., [79]). For both MHC-I AND MHC-II binding peptides, RANKPEP provides a position-specific score matrix (Reche et al., [99]). MHCnuggets is a neural network model based on MHC binders that have been trained on common and rare alleles (Shao et al., [100]). Lopez-Rincon et al. [101] proposed a CNN to classify 553 genome sequences with promising accuracy results for analyzing COVID-19 gene sequences. By giving a wide range of T cell epitopes, Monte Carlo-based simulation has been applied to forecast blueprinting for SARS-CoV-2 vaccines (Malone et al., [102]). It has been documented that the neural network method, NetMHC, predicts which peptides will bind and hence identify epitopes for the SARS-CoV-2 vaccine (Prachar et al., [103]). The application of AI in the research of vaccines and COVID-19 treatment is gaining a lot of attention due to international projects such as CoronaDB-AI, a data collection with genomic features that can be used to train AI models for COVID-19 treatments (KeshavarziArshadi et al., [104]; Liu et al., [105]).  Figure 5 shows AI-based vaccine development for COVID-19. Recent studies have used hidden Markov models, Monte Carlo-based simulation, and neural network approaches to predict epitopes, the portion of an antigen that might stimulate an immune response, as a potential target in the development of a vaccine (Crooke et al., [106]; Prachar et al., [103]; Malone et al., [102]). A deep learning approach (DeepVacPred) has been used for predicting and designing a multiepitope vaccine that could predict 26 different SARS-CoV-2-spike-protein sequence vaccine components (Yang et al., [83]). Deep convolutional neural networks have proven to be a more reliable alternative for predicting MHC and peptide binding (Han and Kim, [107]). Deep learning autoencoders have shown promise in extracting features of human Leukocyte Antigen (HLA-A), which could be used in the development of a vaccine (Miyake et al., [108]). The network of long short-term memory has also shown some encouraging results. This type of RNN was used to predict epitopes for spikes (Abbasi et al., [109]). Malone et al. [102] used a similar strategy, employing deep learning RNN and simulated spike sequences to discover potential vaccination targets. RNN gave sequences for a protein of interest with a high degree of sequence identity. Malone et al. [102] used BepiPred, IEDB, and NEC Immune Profiler tools to create an epitope map for different HLA alleles and studied the complete SARS-CoV-2 proteome beyond spike, to give a comprehensive vaccine design blueprint for SARS-CoV-2. For the development of a vaccine for COVID-19, NLP models, notably language modeling techniques, have made a great impact. Pretrained transformers were utilized in carbohydrate chemistry to predict protein interaction (Nambiar et al., [110]) and model molecular processes (Abbasi et al., [109]), which can be applied in the vaccine development process. The transformers were employed to repurpose commercially available medications by anticipating their interactions with SARS-CoV-2 viral proteins (Beck et al., [111]). Researchers at the University of Basel in Switzerland utilized a protein-modeling tool called the Swiss Model to anticipate the architectures of proteins on the outer surface of the SARS-CoV-2 virus when the pandemic struck. DeepMind, a London-based AI firm, used its AlphaFold neural network to predict the three-dimensional form of SARS-CoV-2 proteins based on the virus's genomic code (Waltz, [49]). Their predictions turned out to be accurate when compared to the virus's actual protein structures.  Table 2 shows some of the common tools for the prediction of epitopes and their evaluated accuracy or reported accuracy, if available.

Therefore, the AI-powered technology offered a ray of hope by assisting scientists and medical health providers in dealing with this deadly disease. To summarize the role of AI in research, AI helps in gathering and synthesizing the information, determining the cause of the disease, and selecting and developing potential drug/vaccine candidates. Furthermore, after the selection of a potential candidate, AI helps in clinical trials of the vaccine.

## 5. AI in Clinical Trials of the Vaccine

The most time-consuming aspect of vaccine research and development is the testing of a vaccine. To acquire a better knowledge of the disease and for the research of a potential vaccine candidate and accelerate its speed, computational approaches and AI techniques have been developed as shown in Figure 6. Several applications of AI help in the rapid classification of novel viruses by detecting their intrinsic genomic structures and can be used to recognize similarities with other pathogens (Randhawa et al., [117]). Only one out of ten molecules get approved for entering into the clinical trials, which is a huge loss for the industry (Hay et al., [118]). The reason for these failures can be caused by a lack of technical needs or infrastructure and poor patient selection. However, with a large amount of digital medical data available, AI can help in reducing these failures (Harrer et al., [119]). Moreover, different AI algorithms help in identifying the potential candidate for clinical trials of the vaccine in an efficient time after the screening of several candidates. Some researchers applied SDQ for reviewing the data of clinical trials in less than 24 hours for the same type of evaluation instead of more than 30 days. The rapid data access was accompanied by exceptional levels of good data quality resulting in a dependable outcome. As a result, the time between molecules to market was reduced from ten years to one year (Kulkarni et al., [120]). After the research for a novel vaccine candidate, it has to undergo a development process. The process is divided into preclinical and clinical trials by regulatory bodies all around the world (Singh and Mehta, [121]). The World Health Organization (WHO), the US Food and Drug Administration (USFDA), and the European Medicines Agency (EMA) have issued guidelines to plan the clinical development path of a potential vaccine candidate. Each vaccine develops in its way, based on the factors including the type of vaccine (peptide/DNA/RNA/inactivated/live), target population, and disease epidemiology. A vaccine candidate normally undergoes three phases of human development known as clinical trials, which are Phase I, Phase II, and Phase III trials before regulatory approval. To monitor the safety and efficacy in the population Phase IV trial is used after the completion of Phase III trials (Farrington and Miller, [122]; WHO technical report, [123]; Hudgens et al., [124]; Collins, [125]).

### 5.1. Different Phases during Clinical Trials of Vaccine

#### 5.1.1. Phase I (20-80 Subjects)

The phase I trial involves healthy subjects. It consists of the administration of the vaccine to subjects. The aim of this trial is the detection of safety and collection of an immune response. The immunization schedule, model of vaccine administered, and dose are often evaluated (Who technical report, [123]; Hudgens et al., [124]; EMEA, 2005).

#### 5.1.2. Phase II (100-300 Subjects)

After reaching a successful outcome in the phase I trial in terms of both immunogenicity and safety, a vaccine candidate should proceed to phase II clinical evaluation. The goal is to provide more information on safety, immunogenicity, and data on the optimal dose, vaccine preparation, and schedule of the vaccine to be taken up for the phase III confirmatory trial (Artaud et al., [126]).

#### 5.1.3. Phase III (Large-Scale Population, 300-3000 Subjects)

The effect of a final formulation is assessed in the phase III trial and is very important for the registration and approval of a vaccine to market. Safety and efficacy are the main goals of these trials. If the vaccine's efficacy and safety are demonstrated in the phase III trial, the manufacturer of the vaccine can submit an application to the national regulatory authority for a license and commercialize the product (Singh and Mehta, [121]).

#### 5.1.4. Phase IV (Several Thousand People)

It is also known as postmarketing surveillance studies (PMS). This trial is used to continue to monitor the vaccine for safety and effectiveness in the population. It is carried out after the successful completion of phase III trials and following licensure of the product (Singh and Mehta, [121]).

The various vaccine candidates are classified according to the technology used for the vaccine development. The list of a few vaccines with their characteristics, manufacturer name, phase 3 trial data, and efficacy data are presented in Table 3 (Kyriakidis et al., [127]).

The majority of the work turns to testing once a vaccine candidate has been designed and developed. Vaccines are initially evaluated in the lab on cells and animals known as preclinical trials, then on human beings known as clinical trials. Unfortunately, AI tools cannot take the place of those time-consuming procedures. However, by applying patient-specific genome-exposome profile analysis, AI can help choose only a certain diseased population for engagement in Phase II and III clinical trials, allowing for early prediction of the viable therapeutic targets in the chosen patients (Mak and Pichika, [128]; Harrer et al., [119]). Predicting lead compounds and preclinical discovery of molecules before the start of clinical trials using AI tools such as predictive ML aid in the early prediction of lead molecules that will pass clinical trials with a selected population of the patient (Harrer et al., [119]). AiCure helps in monitoring the regular medication intake by patients with schizophrenia in phase II trials, resulting in a 25% increase in patient adherence and ensuring the clinical trial's success (Mak and Pichika, [128]). NLP can help in extracting and analyzing important data from patients' EHR records, can compare it to eligibility criteria for ongoing trials, and suggests matching studies. AI tools might be able to forecast which antigens the immune system will encounter, but what the immune system will do in a live human is beyond today's computer capabilities. Because the human body is so complex, AI tools cannot predict what the vaccine candidate will do for the body with reliable data. However, there was no evidence found that clinical trials were conducted using computational supervision. Although AI cannot anticipate the outcome of clinical trials, it can make sense of the mountains of data generated by these trials by analyzing all the factors and identifying patterns that a human brain might miss. As thousands of patients will be engaged as the vaccine candidate progress to the second and third phases of clinical testing, AI tools or systems will be very much critical in quickly assessing clinical and immunological data (Waltz, [49]; Piccialli et al., [129]). To summarize the role of AI in clinical development, it helps in trial planning, optimizing the recruitment process, risk monitoring, toxicity prediction, and also monitoring of drug adherence.

## 6. Conclusion

This paper summarized the application of AI/ML in the field of research and development of the SARS-COV-2 vaccines. AI has been shown as an emerging and promising technology for detecting early coronavirus infection and monitoring the state of affected individuals. AI techniques including ML and DL have shown to be beneficial to aid in the study of the virus by examining the data available and assisting in the development of proper treatment regimens as well as in the development of a novel vaccine candidate. The AI algorithms have become more important for advanced analysis and translation of basic discoveries into novel vaccine candidates due to the large accessible amount of data. However, AI approaches cannot replace the time taking tasks such as laboratory experimentations and clinical trials, but they can aid in the planning of a trial, monitoring, and predictions of deleterious and risk factors. This paper suggested the various computational tools and techniques developed based on AI and ML which can anticipate complicated immune system activities, such as B cell and T cell epitope prediction. With the help of computer-based tools and algorithms, it considerably improves decision-making, and treatment uniformity, and resulted in the speedup in vaccine development and research to fight against the SARS-COV-2 virus.

## Figures and Tables

**Figure 1:** History and evolution of vaccine development by Hilleman.

**Figure 2:** Subbranches of artificial intelligence.

**Figure 3:** (a) Schematic representation of adaptive immunity targeting pathogen for killing. (b) Role of a vaccine in preventing the spread of a virus.

**Figure 4:** Process of vaccine discovery by AI/ML method.

**Figure 5:** AI-based vaccine development for COVID-19.

**Figure 6:** Benefits of employing computational methodologies in vaccine development. The bottom box outlines the points of view and issues raised at each stage of the proposed computational design tools. Processes connected with reverse vaccinology are shown in orange boxes at the bottom.

**Table 1:** Implications of AI/ML in some of the COVID-19 vaccines.

S. No.	Vaccines with manufacturer	Use of AI/ML	References
1.	AZD1222/Covishield AstraZeneca/Oxford University	Used graphical-based knowledge and image analysis to get new clues into illnesses and detect biomarkers 30 percent faster than human pathologists. ML techniques were recently used by AstraZeneca in pathology to speed up the assessment of tissue samples. With the use of big data analysis, AstraZeneca makes it much easier to mine electronic health records (EHR) to optimize clinical trial patient recognition and recruitment. ML and AI were already being used during clinical trials for event assessment to improve the process at various stages with the goal of lowering total duration. ML and AI were already being used during clinical trials for event assessment to improve the process at various stages with the goal of lowering total duration. IoT based on sensor technology came into use that allows for continuous real-time data monitoring and can help to ensure a reliable storage system. If the temperature changes, the sensors will detect it and issue a device alert for the next vaccination shipment.	Weatherall, [68], Kumar and Veer, [65], Sachdeva, [69]

2	mRNA-1273 Moderna	To aid in the designing of mRNA sequences, Moderna employs AI. They went from manually creating roughly 30 mRNAs (a molecule essential to the vaccination) per month to being able to generate almost 1,000 per month because of AI algorithms and robotic automation.	Gast, [63]

3	BNT162b2/Comirnaty BioNTech/Pfizer/Fosum Pharma	Clinical trial data of the COVID-19 vaccine was open to being evaluated 22 hours after reaching the primary efficacy cases counts, due to Pfizer's new ML technology, SDQ. Using the technology, the team was able to maintain a high level of data value throughout the trial, with just minor differences to fix in the latter stages. They used AI and MI to forecast product throughput and yield, which enables for more consistent production and predictability in our manufacturing, which is critical given the urgency of ramping up our vaccine production. The company utilized ML and AI to anticipate product temperatures and enable preventative maintenance for the over 3,000 freezers that store our vaccine doses, and we employ IoT and sensors to track and monitor vaccine deliveries and temperatures with near-perfect precision. Supercomputing was used to run molecular dynamics simulations to determine the best mix of lipid nanoparticle features for reducing allergic responses, resulting in a vaccination that is both safe and effective. To manage patient reporting more efficiently throughout clinical trials, the business introduced an upgraded adverse event portal with AI capabilities.	Peckham, [70]

4.	BBV152/Covaxin Bharat Biotech	A storage temperature of 2–8°C is required. Hence, IoT based on sensor technology came into use that allows for continuous real-time data monitoring and can help to ensure a reliable storage system. If the temperature changes, the sensors will detect it and issue a device alert for the next vaccination shipment.	Kumar and Veer, [65], Sachdeva, [69]

**Table 2:** Some tools for the prediction of epitopes.

Technique	Method	References
RANKPEP	Prediction of MHC binding peptides, for MHC-I accuracy, is 80% and MHC-II is 0.96 AUC	He et al., [112]; Yazdani et al., [113]
MHCnuggets	A neural network (LSTM) model based on MHC binders that have been trained on common and rare alleles and self-reported accuracy of 0.924 AUC	Campbell et al., [114]
NetCTLpan1.1	Prediction tool for MHC-I epitopes and self-reported accuracy of 0.976 AUC	Ayyagari et al., [87]; Mishra et al., [86]; Safavi et al., [115]
BepiPred (2.0)	RF-based and ML-based models trained on epitopes and self-reported accuracy of 0.62 AUC	Rahman et al., [116]; Ayyagari et al., [87]; He et al., [112]; Khairkhah et al., [85]
DeepVacPred	Prediction and designing of a multi-epitope vaccine	Yang et al., [83]
IgPred	SVM-based B cell epitope prediction tool can be used to remove candidates with a high resemblance to IgE epitopes	Gupta et al., [84]

**Table 3:** List of a few vaccines with their characteristics, phase 3 trial data, and efficacy data (Kyriakidis et al., [127]).

Vaccine type	Candidate vaccine name	Manufacturer(s)	Phase 3 trial starting date	Number of participants	Antibody response rate	Clinical trial registration number	Efficacy	Beneficial features
Replication-defective viral vector vaccine	(1) Ad5-nCoV (2) AZD1222 (3) Sputnik V/Gam-COVID-Vac (4) JNJ-78436735/Ad26.COV2.S	(1) CanSino Biological/Beijing Institute of Biotechnology/Academy of Military Medical Sciences (2) AstraZeneca/Oxford University (3) Gamaleya Research Institute/Health Ministry of Russian Federation/Acellena Contract Drug Research and Development (4) Janssen Pharmaceutical Companies of Johnson & Johnson/Beth Israel Deaconess Medical Center	(1) September, 2020 (2) August, 2020 (3) September 7, 2020 (4) September 23, 2020	(1) 40,000 (2) 30,000 (3) 40,000 (4) 90,000	(1) Neutralizing antibodies produced in 97% of the participants (Phase 2) (2) Neutralizing antibodies produced in all participants that received the prime-boost regime (Phase 1/2) (3) Neutralizing antibodies produced in all participate (Phase 1/2) (4) Neutralizing antibodies in 92% of the participants (Phase 1/2a)	(1) NCT04526990 (2) NCT04516746 (3) NCT04530396 (4) NCT04614948	(1) N/A (2) 62.1% overall and 90% (18 to 55 years old) (3) 91.4% (4) N/A	Can induce robust humoral and cellular responses with a single dose. Good safety profile

mRNA vaccine	(1) mRNA-1273 (2) BNT162b2/Comirnaty	(1) Moderna/NIAID (2) BioNTech/Pfizer/Fosum Pharma	(1) July 27, 2020 (2) July 27, 2020	(1) 30,000 (2) 44,000	(1) Neutralizing antibodies produced in all participants (Phase 1) (2) Neutralizing antibodies produced in all participants (Phase 1)	(1) NCT04470427 (2) NCT04368728	(1) 94.1% (2) 95% overall 94% (>65 years old)	Scalability. Fast design and development. Extremely safe. No infectious agent in handling. Can induce and cellular responses

Protein subunit vaccine	(1) NVX-CoV2373 (2) ZF2001	(1) Novavax (2) Longcom/Chinese Academy of Medicine	(1) September 23, 2020 (2) November 18, 2020	(1) 45,000 (2) 29,000	(1) High titers of neutralizing antibodies in all participants (Phase 1/2) (2) Not reported	(1) NCT04511802 (2) NCT04646590	(1) N/A (2) N/A	Safety during production. Can be safely administered to immunosuppressed people. No infectious agent handling is required

Inactivated pathogen vaccine	(1) CoronaVac (2) Undisclosed (3) BBIBP-CorV (4) BBV152/Covaxin	(1) Sinovac Research and Development Co. (2) Wuhan Institute of Biological Products/China National Pharmaceutical Group-Sinopharm (3) Beijing Institute of Biotechnology/China National Pharmaceutical Group-Sinopharm (4) Bharat Biotech	(1) July 21, 2020 (2) July 18, 2020 (3) July 16, 2020 (4) November 16, 2020	(1) 8,870 (2) 21,000 (3) 63,000 (4) 26,000	(1) Neutralizing antibodies in 92.4% and 97.4% of the participants that received two doses of 3 *μ*g of vaccine 2 or 4 weeks apart, respectively (Phase 2) (2) High titers of neutralizing antibodies in all participants that received the higher dose (Phase 1/2) (2) High titers of the neutralizing antibodies in all participants (Phase 1/2) (3) Neutralizing seroconversion rate 93.4% in 3 *μ*g/dose group (Phase 1)	(1) NCT04456595 INA-WXFM0YX (2) ChiCTR2000034780 ChiCTR2000039000 (3) NCT04560881 NCT04510207 ChiCTR2000034780 (4) CTRI/2020/11/028976	(1) N/A (2) N/A (3) 79.34% (4) N/A	Safety, as the pathogen is dead. Transport and storage

Virus-like particles	CoVLP	Medicago/Glaxo Smith Kline	November 19, 2020	30,612	Not reported	NCT04636697	N/A	They combine the efficacy of attenuated vaccine and the safety subunit vaccines. Scalability of production. Their size makes them ideal for uptake by APCs

## Data Availability

No data were used.
